# Non-coding RNAs in cancer: platforms and strategies for investigating the genomic “dark matter”

**DOI:** 10.1186/s13046-020-01622-x

**Published:** 2020-06-20

**Authors:** Katia Grillone, Caterina Riillo, Francesca Scionti, Roberta Rocca, Giuseppe Tradigo, Pietro Hiram Guzzi, Stefano Alcaro, Maria Teresa Di Martino, Pierosandro Tagliaferri, Pierfrancesco Tassone

**Affiliations:** 1 Laboratory of Translational Medical Oncology, Department of Experimental and Clinical Medicine, Magna Graecia University, Salvatore Venuta University Campus, 88100 Catanzaro, Italy; 2 Medical and Translational Oncology Units, AOU Mater Domini, 88100 Catanzaro, Italy; 3 Net4science srl, Magna Graecia University, Salvatore Venuta University Campus, 88100 Catanzaro, Italy; 4 Laboratory of Bioinformatics, Department of Medical and Surgical Sciences, Magna Graecia University, Salvatore Venuta University Campus, 88100 Catanzaro, Italy; 5 Department of Health Sciences, Magna Græcia University, Salvatore Venuta University Campus, 88100 Catanzaro, Italy

**Keywords:** Cancer genetics, Non-coding RNAs, microRNAs, miRNAs, Long-non coding RNAs, lncRNAs, ncRNA functions

## Abstract

The discovery of the role of non-coding RNAs (ncRNAs) in the onset and progression of malignancies is a promising frontier of cancer genetics. It is clear that ncRNAs are candidates for therapeutic intervention, since they may act as biomarkers or key regulators of cancer gene network. Recently, profiling and sequencing of ncRNAs disclosed deep deregulation in human cancers mostly due to aberrant mechanisms of ncRNAs biogenesis, such as amplification, deletion, abnormal epigenetic or transcriptional regulation. Although dysregulated ncRNAs may promote hallmarks of cancer as oncogenes or antagonize them as tumor suppressors, the mechanisms behind these events remain to be clarified. The development of new bioinformatic tools as well as novel molecular technologies is a challenging opportunity to disclose the role of the “dark matter” of the genome. In this review, we focus on currently available platforms, computational analyses and experimental strategies to investigate ncRNAs in cancer. We highlight the differences among experimental approaches aimed to dissect miRNAs and lncRNAs, which are the most studied ncRNAs. These two classes indeed need different investigation taking into account their intrinsic characteristics, such as length, structures and also the interacting molecules. Finally, we discuss the relevance of ncRNAs in clinical practice by considering promises and challenges behind the bench to bedside translation.

## Background

Carcinogenesis is a multistep process in which normal cells acquire genetic and epigenetic alterations that drive the onset of “hallmarks” of cancer finally resulting in development and progression of malignancies [1]. Despite most cancer studies have been focused on protein-coding genes, the evidence that about 97% of human genome consists of non protein-coding sequences led scientists to investigate this genetic “dark matter” in tumorigenesis. The untranslated transcripts, called non-coding RNAs (ncRNAs) can be classified in short (19–31 nucleotides), mid (20–200 nucleotides) and long (> 200 nucleotides) based on their length. Among them, the most extensively studied in cancer are micro-RNAs (miRNAs), which belong to short ncRNAs class (22–25 nucleotides in length) [2] and long-ncRNAs (lncRNAs), which represent the largest class of non-coding transcripts with about 55,000 genes along the human genome [3]. According to miRNA-mRNA complementarity, miRNAs can mediate post-transcriptional gene regulation by translational repression or mRNA degradation, while lncRNAs may regulate gene expression through their interaction domains for DNA, mRNAs, miRNAs and proteins. These events are dependent from both their sequence and secondary structure [4]. Specifically, ncRNAs can affect cancer cell fate and survival through a variety of different mechanisms, including transcriptional and post-transcriptional modification, chromatin remodeling and signal transduction. However, to date the exact function and mechanism of action of most of them is still unknown. As far as we know, ncRNAs create a complex network of mutual interactions [5] and act as oncogenes or tumor suppressors. They present a tissue specific expression pattern, which is highly dysregulated in cancer, and are considered promising diagnostic, prognostic and therapeutic targets [6–8]. Therefore, the understanding of the role of ncRNAs in tumorigenesis is a challenging goal in current biology. In this review we describe the in silico and in vitro approaches aimed to investigate the ncRNA transcriptome by providing a comprehensive overview of strategies and tools to characterize ncRNA structure and to study their contribution in cancer onset and progression (Fig. 1). Moreover we underline the promises and limits of these approaches in terms of translational relevance.

**Fig. 1:** Schematic representation of the approaches discussed in this review for the investigation of the role of ncRNAs in human cancer

## NcRNAs expression profiling

The aberrant expression of ncRNAs is an important feature of human cancer [9–11]. The ncRNAs have cell type, tissue and cancer specificity, thus RNA profiling has become a mean to identify useful biomarkers of tumor development, progression and metastasis. Although miRNAs represent the most widely investigated ncRNAs, lncRNAs are emerging as cancer key regulators [7, 12]. Arrays and next generation sequencing (NGS) are high-throughput methods to detect and quantify ncRNAs, even though several caveats are to be considered. Typically, both miRNAs and lncRNA are expressed at lower abundance if compared to mRNAs (~ 0.01% and ~ 0.1% of total RNA, respectively) [13]. In particular, miRNA profiling requires RNA isolation procedures to retain the small RNA fraction. In addition, miRNAs lack a common sequence, such as poly(A) tail, that is typically observed in mRNAs, so it is necessary to selectively detect this class of ncRNAs among different RNA species. Moreover, miRNAs of the same family may show high similarity or differ from the reference sequence due to post-transcriptional modifications (isomiRs). In contrast, lncRNAs have similarities with mRNAs such as size, RNA polymerase II transcription, 5′-capping, RNA splicing, and also about 60% of lncRNAs include a poly(A) tail. For this reason, lncRNAs can be profiled together with mRNAs while miRNAs require different approaches. However, the design of probes for many lncRNAs is difficult because most lncRNAs are located at intergenic regions with high GC content or are antisense transcripts of known protein coding genes. Here we report various methodologies to investigate differences in the pattern of gene expression between normal vs cancer cell, in order to discover ncRNAs potentially involved in tumorigenesis [14].

### Microarray

Microarray is a well-established method to profile both miRNAs and lncRNAs, although it was initially designed for protein-coding mRNAs. This technology is based on nucleic acid hybridization between labeled RNA targets and their specific and complementary probes. Advantages of microarrays are the high parallel analysis coupled with relative cost and the ability to detect low levels of molecules of RNAs without the need of PCR-enrichment steps. Various platforms for miRNA profiling include different direct miRNA labelling procedures without amplification. LncRNA microarray platforms systematically profile lncRNAs together with mRNAs. Generally, lncRNA platforms include an in vitro transcription (IVT)-based amplification step and are characterized by less technical variations respect to miRNA platforms and mainly differ for the number of lncRNAs analyzed. For example, the *Agilent SurePrint G3 Gene Expression v3 microarray*, targeting 30,606 human lncRNA transcripts, covers all of LNCipedia 2.1, the *Arraystar LncRNA microarray* (release Human v5.0) profiles 39,317 lncRNAs, *Clariom D human array* from Thermo Fisher Scientific covers more than 55,900 lncRNA NONCODE transcripts. Limitations of microarrays for ncRNA analysis are a restricted linear range of quantification, the design of probes limited to known sequences, the need for continuous updating of annotations, the relative quantification limited to compare different status (for example, healthy versus affected). An example of microarray technology application has been reported by Zhou et al. which profiled 389 colon cancer patients identifying a signature of six lncRNAs (linc0184, AC105243.1, LOC101928168, ILF3-AS1, mir31HG, and AC006329.1) associated to risk of cancer recurrence [15], or by Liang et al., which identified through this technology, six miRNAs involved in breast cancer pathogenesis (hsa-miR-21b, hsa-miR-29b, and hsa-miR-155 as upregulated and hsa-miR-10b, hsa-miR-125 and hsa-miR-145 as downregulated) [16]. Another technique based on microarray is the Tiling array that differs because of the use of probes that may cover either specific chromosomal sequences as well as contiguous regions or even the whole genome. Bertone et al. found 10.595 transcribed sequences not detected with other methods in 2004 [17] but in the current biology, this technology has been replaced by NGS approaches.

### Sage

Serial Analysis of Gene Expression (SAGE) is the first high-throughput sequencing technology developed to analyze the transcriptome in term of identification and quantification of transcripts, including ncRNAs [18]. It is based on the restriction enzymes-mediated generation of short-stretches of unbiased cDNAs sequences (9 bp SAGE tags) followed by concatenation, cloning and sequencing. This method has been implemented in the “SuperSAGE” variant that allows the profiling of 26 bp tags and provides the advantage of in tag-to gene annotation by generating more throughput data with a better quality/cost ratio [19]. Gibb et al. reported lncRNA expression profile across 26 normal and 19 tumoral tissues by analyzing 24 million SAGE tags [20].

### RNA-seq

RNA sequencing (RNA-seq) allows the detection and quantification of all classes of ncRNAs through the construction of different cDNA libraries, specific for each type of ncRNA. cDNA library preparation is followed by massive parallel sequencing of transcripts of interest. The small RNA-seq is suitable for the sequencing of small ncRNAs, while total RNA-seq is recommended for lncRNA sequencing as many lncRNAs may not be polyadenilated. Compared to microarray, RNA-seq offers a more comprehensive coverage of whole transcriptomes. Importantly, RNA-seq is design-free probe allowing the detection of unknown/novel transcripts and also the detection of sequences that differ, even for a single nucleotide, such as transcripts harboring mutations or isoforms. The main limitations of RNA-seq are the complexity of data analysis and the high deep reads needed to detect low amount of the target. Using RNA-seq technology Yamada et al. identified a signature of 27 upregulated and 22 downregulated lncRNAs associated with colorectal cancer (CRC) as alternative biomarkers and/or treatment targets [21]. Yu N et al. identified tumor suppressor in lung adenocarcinoma by integrating data from miRNA-seq and RNA-seq [22]. The most advanced application of RNA-seq is the single cell transcriptomic sequencing [23]. For example, Designed Primer-based RNA-sequencing strategy (DP-seq) allows the amplification of RNA from 50 pg of sample [24], while Quartz-Seq is a single cell RNA seq method able to reveal genetic changes between single cells into the same cell type and also into the same cell-cycle phase [25].

### Cage

Cap analysis gene expression (CAGE) is an NGS-based technology allowing the generation of a snapshot of the 5′ end of the mRNA. Similarly to SAGE, sequencing is preceded by cDNAs-tag generation, concatenation and cloning, but the main differences between the two approaches is the ability of CAGE to identify the exact location of the 5′ capped- transcript. Respect from RNA-seq, the advantage of CAGE consists in the identification of transcriptionally active promoter regions and RNA polymerase II transcription start sites (TSS). Horie et al. revealed a set of 49 coding and 10 non-coding genes upregulated in non-small cell lung cancer (NSCLC) due to promoter hypomethylation, by performing an integrative analysis of promoter level expression profiles generated through CAGE method [26].

## In silico investigation

High-throughput ncRNAs expression profiling methods require bioinformatic contribution to analyze data generated from different platforms, including microarray and NGS technologies described above. In particular, the application of NGS is becoming predominant to explore in depth patient specific genetic background underlying intra and inter-individual variability, which acquire increasing relevance in the era of personalized medicine [27–30]. Analysis of ncRNAs data may have different aims such as discovery and annotation of novel ncRNAs, expression pattern profiling, validation and structural reconstruction of known ncRNAs and integrative analysis of their behavior and functions.

### Bioinformatic analysis

In the case of data generated by array technology, bioinformatic data analysis includes: *i)* the identification of differentially expressed genes between two classes (such as normal versus tumor specimens, pharmacological treated versus non-treated cells, etc.), *ii)* clustering, which consists in building clusters of genes in term of expression level, *iii)* classification and/or, *iv)* analysis of pathways and interaction networks. Microarray raw data processing involves 4 phases: 1) pre-processing, which includes background adjustment, normalization and summarization, 2) annotation to enrich preprocessed data, 3) statistical and/or data mining analysis and 4) biological interpretation. Well-known algorithms of microarray data preprocessing are MAS4.0, MAS5.0, RMA, PLIER and GCRMA. Background correction is essential to remove noise in the optical detection system due to non-specific hybridization. Normalization, within and between arrays, is needed in order to remove systematic technical artifacts that could be due to different efficiency of reverse transcription, labeling or hybridization reactions, or other laboratory conditions. Summarization unifies signals generated from multiple probes, designed for the same transcripts, with multiple locations on the array. Once summarized, data can be annotated by adding information such as gene symbols or function. Data mining is the process by which groups of samples are compared in order to find differentially expressed genes on the basis of their expression values. Many of the methods for visualization and interpretation of gene expression data can be used for both microarray and RNA-seq experiment including clustering analysis, gene set enrichment analysis and pathway (Gene Ontology, KEGG, Ingenuity, Reactome, WikiPathways) or network analysis [31, 32].

In the case of RNA-seq, ncRNAs analysis workflow starts from raw NGS data. The first step is the filtering of low-quality reads from raw data. This process is usually performed by using tools for pre-processing of files containing short-reads encoded into FASTA-FASTQ files, which map the sequences to reference data (stored into databases). Example of such programs are the FASTX-Toolkit, Blat, SHRiMP, LastZ, MAQ and many others [33]. Once filtered, the second step is to construct transcript assembly using, for instance BowTie [34] or TopHat [35]. After the assembly, known genomic sequences, i.e. known coding genes, are filtered by tools, such as Bowtie. At the end of this step all the sequences may represent potential noncoding RNAs that have to be assessed and mapped with respect to existing ncRNA databases using assessment tools such as CPAT or Pfamscan. The NCBI NT and NR database is the preferred mapping database in this step since they include sequences for all species. NcRNAs extraction from RNA-seq and assembled transcripts processing can be instead performed by using many different approaches, many of which implement sequential filters based on features such as transcripts length, number of exons for each identified transcript or Open Reading Frame (ORF) size. Sun et al. presented a pipeline called lncRNAscan able to detect novel lncRNAs from the transcripts file generated by RNA sequencing [36]. Machine learning based algorithms and comparative sequence analysis have also been investigated in literature [37–39]. The above described pipeline is used in almost all the bioinformatic studies related to ncRNAs [2, 5, 40, 41] in which ncRNAs expression pattern has been correlated with clinical outcome of cancer patients. Finally the function of ncRNAs has to be investigated by analyzing existing databases (summarized in Table 1) hosting a large number of ncRNA sequences and, when available, information about biological studies. These databases can be queried to identify known ncRNAs in a given dataset but, due to the lack of conservation, many known ncRNAs are only valid for well-annotated species. For example, Song et al. [42] used the lnRNAdb to support the identification of lncRNAs with a potential role in human gastric cancer occurrence and development. Hou et al. used NONCODE database to detect coding and noncoding genes extracted from cell RNA-seq data and bulk hepatocellular carcinomas cells data [43].

**Table 1:** Summary table of the most popular databases and tools storing information about micro and long ncRNAs

DATABASE and TOOLS	BRIEF DESCRIPTION	LINK	AVAILABILITY	PROS (+)/CONS (−)
**NONCODE**	Contains a total of 487.164 lncRNA transcripts and 324.646 lncRNAs genes for 16 different species and allows searching sequences, expression, orthologs, functions and diseases related, to a given input gene or transcript.	http://www.noncode.org/	PA	(+) High Number of sequences (+) 17 different species (+) Disease Association (+) Simple Analysis (+) High level of manual curation
**LncRNAMap**	Is a web resource for studying lncRNAs in the human genome and currently contains 23.355 lncRNAs with sequences retrieved from Ensembl 65 (GRCH37)	http://lncrnamap.mbc.nctu.edu.tw/php/	PA	(−) No Analytic potential (−) No recent updates
**LNCipedia**	Includes 127.802 human lncRNAs transcripts, provides sequence, annotations and manually curated lncRNA articles	https://lncipedia.org/	PA	(+) Recent Web Interface (+) API Interface for data integration (+) Submission of novel sequences
**LncRNADisease**	Integrates approximately 1000 lncRNAs-to-disease associations, including cancer, obtained using lncRNA -disease prediction tools that compare lncRNA genomic location with the closer gene	http://www.cuilab.cn/lncrnadisease	PA	(+) Prediction of associations on the basis of user-provided sequences (+) High level of manual curation (+) Submission of novel sequences (−) Web Interface Obsolete
**lncRNAdb**	Is a database of long-noncoding RNAs in eukaryotes storing both raw data about sequence as well as other referenced information such as structural information, genomic context, levels of expression, and functional information	https://rnacentral.org/expert-database/lncrnadb	PA	(−) Limited number of sequences (+) Extensive annotation and biological knowledge is provided (+) High level of manual curation
**LncRNA2Target**	Expression profiling analysis following lncRNA Knockdown or Overexpression	http://123.59.132.21/lncrna2target/	PA	(−) Limited Scope (−) Obsolete web interface
**NRED**	Provides comprehensive information on lncRNAs and lncRNA expression data from microarray and In situ Hybridization data	https://www.hsls.pitt.edu/obrc/index.php?page=URL1237993821	PA	(−) Limited Scope (−) Obsolete web interface
**GENCODE**	Contains ncRNA gene annotations in .gtf format and ncRNA transcript sequences in .fasta format. Its goal is the investigation of gene features based on biological evidence	https://www.gencodegenes.org/	PA	(−) Limited access (only by FTP) (−) Limited Query Capabilities
**ENCORI**	Is focused on miRNA-target interaction, including miRNA-lncRNA and protein-lncRNA interaction data	http://starbase.sysu.edu.cn/	Upon Request	(−) No Simple Access
**NPInter**	Stores functional interactions between ncRNAs and other molecules (DNAs, RNAs and proteins) and is regularly updated with novel interactions coming from manual curation of literature, high throughput screening and in silico predictions.	https://omictools.com/npinter-tool	PA	(+) Regular Updating (+) High level of manual curation
**DIANA TOOLS**	Is a tool for determining miRNA and lncRNA interaction based on experimental studies and computational prediction	http://carolina.imis.athena-innovation.gr/diana_tools/web/index.php?r=lncbasev2%2Findex	PA	(+) Prediction of Interactions (−) Limited number of stored information on interactions
**GeneCards**	Provides comprehensive information about coding and non coding genes	https://www.genecards.org/	PA	(−) No Analytic Capabilities
**SomamiR**	Includes information about somatic mutations in miRNA or miRNA-target site sequences and on biological pathways affected by these alterations	http://compbio.uthsc.edu/SomamiR/	PA	(+) Somatic Information
**PROGmiR**	Give information about the potential role of miRNAs as cancer biomarker	https://omictools.com/progmir-tool	PA	(+) Highly Tailored for cancer (−) No information for other diseases
**miRCancer**	Contain data about miRNA-cancer association obtained through data mining	http://mircancer.ecu.edu	PA	(+) Highly Tailored for cancer (−) No information for other diseases
**miRBase**	Includes published miRNA sequence and annotation, available for download	http://www.mirbase.org/index.shtml	PA	(+) Highly Tailored for cancer (−) No information for other diseases
**miRwalk**	Provides information about miRNA-target interaction	http://zmf.umm.uni-heidelberg.de/apps/zmf/mirwalk2/	PA	(+) High potential for custom analysis
**miRDB**	microRNA target prediction tools	http://mirdb.org/	PA	(−) Limited Analysis
**TargetScan**		http://www.targetscan.org/vert_72/	PA	(+) High potential for custom analysis
**miRTar.human**		http://mirtar.mbc.nctu.edu.tw/human/	PA	(+) Possibility of downloading and use in local for batch analysis
**miRmap**		https://mirmap.ezlab.org/	PA	(+) High potential for custom analysis
**miRDeep2**	microRNA deep sequencing tools	http://ibis.tau.ac.il/miRNAkey/	PA	(−) Not user friendy (−) Requires programming skills (−) No recent updates
**miRNAkey**		https://bio.tools/mirnakey	PA	(−) Not user friendy (−) Requires programming skills - No recent updates

*PA* Public Available

### Computational biology prediction

In the context of the investigation and discovery of ncRNAs involved in cancer cell biology, it is important to identify and predict such molecules by computational methods. Therefore, several algorithms have been developed or used for accurate and fast prediction of ncRNAs, with the aim to avoid expensive experimental methods [44]. Notwithstanding, the accuracy of these algorithms is reduced by increasing ncRNA nucleotide sequence length, thus lncRNAs prediction suffers from numerous limitations and approximations, while miRNAs are more easy to be modelled. The algorithms development for predicting ncRNAs requires specific models [45], among them *i)* Minimal Folding Energy (MFE), *ii)* Hidden Markov Model (HMM) and *iii)* Stochastic Context Free Grammar (SCFG), whose application led to the reconstruction of the 2D structure of ncRNAs (Fig. 2). MFE is an RNA structure-based model that considers base pairs and their related energy. Therefore, by applying the canonical base pairing between A-U, C-G and the unusual G-U [46, 47] together with thermodynamic laws [48], the structure showing the lowest energy is selected as the most stable. However, the MFE predictions are based on different assumptions about native RNA structures and suffer some limitations, which enable MFE to identifies ~ 70% of bp correctly for RNAs under ~ 700 nt in length, only [49]. Among MFE based algorithms RNAfold, RNAstructure and Mfold have been widely used to predict 2D structure of ncRNAs. For example, Rahimi et al. explored potential hairpin structures and differentiated real miRNA precursors from pseudo ones through the application of RNAfold, allowing the selection of hsa-miR-B43 as one of the best candidates which might have a potential metastasis-related function in breast cancer [50]. RNAfold and RNAstructure were also able to demonstrate that the free energy of miR-302c stem-loop structure was more negative in the presence of the wild-type compared to the variant allele, leading to the suggestion that rs199971565 SNP is a novel INDEL biomarker located in the seed site of miR-302c, which may have crucial roles in the susceptibility to gastric cancer [51]. HMM is a probabilistic model and belongs to methods able to find similarity between sequences. BLAST and FASTA algorithms are considered the easiest methods, which can determine sequences similarity between homologous families [52]. HMM is to be preferred in the case where sequence similarity between distant families is required. Thus, it is useful to identify the most likely positions containing ncRNAs sequences. In particular, the similarity between query sequence and the consensus sequences is established through the alignment employing the constructed scoring matrix. Vorozheykin et al. applied this model in a web server for prediction of pre-miRNAs, miRNAs, and their binding sites [53]. Voss et al. developed RNAlishapes [54]: an ab initio algorithm able to predict ncRNA genes applying HMM method. In particular, it predicts ncRNAs through the identification of transcription start points or other unique positions in a genome. Finally, SCFG is a statistical method capable of modeling interactions between base pairs in the structure of RNA and is used to predict structure and sequence of ncRNAs. As HMM extends regular grammars, SCFGs extends context-free grammars in which each production is attached to a probability. Simply, ncRNA secondary structures are assimilated to symbols and the comparison of similarity between target sequences and such symbols can predict most likely sequences as ncRNAs. In this model, the dynamic programming algorithm detects secondary structures with the maximum score for their functions. Two important algorithms, that use this model, are Rfam and tRNAscan [55].

**Fig. 2:** Three of the most important models required for the development of algorithms predicting 2D ncRNAs: Minimal Folding Energy (MFE), Hidden Markov Model (HMM) and Stochastic Context Free Grammar (SCFG)

Computational techniques are also useful in the identification of ligands interacting with lncRNA. In this field, a useful software is Inforna. It is able to predict motifs (secondary structures) within the target and drives sequence-based design of small molecules (SMs) targeting structured RNAs [56]. Recent studies also demonstrated the suitability of classical computational methods, such as docking and molecular dynamics, by working on lncRNA 3D structures, thanks to the target of discrete binding pockets in nucleic acids [57, 58] (Fig. 3). Unfortunately, the number of available lncRNA crystallographic structures is still very small, thus making more difficult the identification or the design of specific inhibitors. Currently, the literature reported successful drug discovery studies on three particular lncRNAs: TERRA, MALAT-1 and HOTAIR [59–61].

**Fig. 3:** Possible application of computational biology prediction starting from lncRNAs 3D structure

## Validation of ncRNAs expression

Data obtained from microarray or RNA-seq, as well as from the in silico predictions need hortogonal validation. The evaluation of ncRNAs expression level can be performed through different approaches, such as northern blot (NB), reverse transcription quantitative PCR (RT-qPCR), in situ hybridization (ISH) or fluorescence in situ hybridization (FISH).

### Northern blot analysis

NB analysis is the earliest technique used to analyze gene expression splicing variants of a given ncRNA. The procedure involves the use of gel electrophoresis to separate RNA samples followed by RNA transfer onto a nylon membrane, RNA-probe hybridization and finally RNA-probe detection. An example of the application of this approach has been reported from Vanas et al., which used NB to measure miRNA-21 in osteosarcoma cell lines, by demonstrating that its expression is involved in cell proliferation and regulation of cisplatin activity [62], while Liu J et al. described lncRNA PANDAR as new prognostic and therapeutic target in gastric cancer, on the bases of expression levels [63]. The main limitation of this method is the low sensitivity and the high time consumption. A large amount of total RNA for samples is required and this is very problematic for low-abundant miRNAs or limited cell or tissue source of RNA samples. Moreover, the use of isotope labeling in the classical protocol is hazardous and thus restricted by many institutions. In recent years, several improvements have been made to the classical method using non-radioactive labeling such as digoxigenin (DIG)-labeled modified probes [64]. Probes have been modified with locked nucleic acid (LNA) structure or biotin to increase affinity and sensitivity [65].

### Reverse transcription quantitative PCR

The RT-qPCR is one of the most used method of detection and quantification of ncRNAs as easily to be incorporated in laboratory workflow. This method is often used to validate data obtained from microarray, as reported i.e. by He et al., which analyzed the differential expression profile of miRNAs in peripheral blood of lung cancer patients [66]. RT-qPCR technique include both TaqMan and SYBR green assays. The reverse transcription step varies on the basis of ncRNA of interest. In TaqMan assay, miRNAs are reverse transcribed using a specific stem loop RT primer, while SYBR green protocol includes the addition of a poly-A tail to miRNA sequence to allow primer binding. For lncRNA reverse transcription is performed using random primers or a specific RT primer followed by qPCR with real-time monitoring of reaction product accumulation using both TaqMan or SYBR green chemistry. Commercially available customizable plates and microfluidic cards can be designed either to examine a small set of ncRNAs or to provide more comprehensive coverage. Using RT-qPCR as a quantification method, it has been possible to demonstrate that the lncRNA HOTAIR is an independent predictor of metastatic spread and death in breast cancer patients [67].

### In situ hybridization and fluorescence in situ hybridization

In recent years, advances in probe technologies and detection methods have improved ncRNA visualization by the application of ISH and FISH methods, based on the use of fluorescent probes binding the nucleic acid sequence presenting the highest degree of complementarity. FISH and ISH provide information regarding the spatial-temporal expression of ncRNAs and their subcellular localization providing novel information on ncRNA biological function. For example, confocal microscopy for FISH demonstrated that lncRNA NKILA exerts its critical function in cellular cytoplasm preventing NF-κB activation through stabilization of NF-κB/IκB complex by playing an essential role in turning off cancer-associated inflammation [68]; while ISH method applied to miRNAs allowed the identification of miR-375 downregulation as prognostic factor of esophageal squamous cell carcinoma [69]. The use of fluorophore-labeled DNA or RNA probes methods, is highly challenging due to the short length and the presence of repetitive sequence. Examples are the application of fluorophore-labeled multiple oligo probe sets [70], LNA probes [71] and branched-DNA probes [72]. The use of modified oligonucleotides, such as LNA or 2′-O-methyl (2OMe) [73] has significantly increased specificity and affinity to RNA targets. In particular, the use of hapten-labeled LNA oligos has been found to be highly advantageous in the detection of miRNAs in experimental and clinical tissue samples [74] whereas only a few reports are published for lncRNAs detection [75]. To overcome the limitations of these methods to detect low abundance of ncRNAs, researchers have developed and applied single-molecule RNA FISH based on hybridization of multiple short fluorescently labeled oligonucleotide of a single cell [76]. The use of a single oligo probe, optimally designed and with minimum cross-binding to other RNAs, reduces the risk of off-target probe hybridization.

## Investigation of ncRNAs interactome

Non-coding RNAs exert their functions by direct interaction with other partners, which could be RNA in the case of miRNAs, and RNA, DNA and/or proteins in the case of lncRNAs.

In a previous manuscript we discussed about the integration of multi-omics data from different molecular levels in order to underline the complexity of the biological interactions. In that context we mentioned integrative analyses performed between transcriptomic data (e.g. miRNA and mRNA expression) together with genomics and epigenomics data (e.g. methylation profiling) to highlight the functional interactions between coding and non coding genes [77]. Here, we afford to point out the networks involving lncRNAs, miRNAs and coding genes in terms of cooperation and reciprocal regulation in the biological pathways which have a driver role in human cancer. The molecular mechanisms behind these interactions have been described, even tough technological advances allow the continuous updating and refinement of the understanding of these molecular events [78, 79]. MiRNAs work as negative regulators of coding transcripts by direct binding to mRNA. On the other hands, lncRNAs modulate the biologicial pathways through various mechanism at genomic, trascriptional and post-trascriptional level such as *i)* chromatin remodeling through histone modifications, *ii)* recruitment of transcription factors, *iii)* RNA polymerase II binding, iv) alternative splicing, v) mRNA stability, vi) recruitment of polysomes, vii) gene expression regulation in neighbor cells through extracellular vesicles and viii) miRNA interaction [80]. For what concerns the lncRNA-miRNA direct post-trascriptional interaction, 4 different mechanisms have been proposed: *i)* miRNA-triggered lncRNA decay, in which lncRNA degradation is induced by miRNA binding *ii)* lncRNA acting as miRNA sponge/decay, in which lncRNAs sequestrate miRNAs by removing their negative control on target mRNA *iii)* lncRNA-miRNA competition for mRNAregulation and *iv)* lncRNA generating miRNAs by alternative splicing [81].

Several studies focusing on non coding-coding genes interactions in human cancer, have been aimed to identify lncRNA-miRNA-mRNA axes which may promote tumor growth. For example Yu Lian et al. identified the role of the oncogenic lncRNA AFAP-AS1 to promote nasopharyngeal carcinoma metastasis by binding miR-423-5p and modulating the RAB11B and LASP1 coding genes involved in the Rho/Rac signaling pathway [82]. Han Li et al. demonstrated a feedback loop in the regulation of the malignant behaviors of glioma cells in which are involved the lncRNA SNHG1, microRNA-154-5p or miR-376b-3p and the coding gene FOXP2. This axis leads to the enhanced expression of KDM5B, which is an RNA-binding protein able increase the stability of SNHG1 [83]. A transcriptomic analysis of mRNA-lncRNA and miRNA interaction, performed by Xia Tang et al., revealed their synergistic network in hepatocellular carcinoma by highlighting the interaction between 16 miRNAs, 3 lncRNAs and 253 mRNAs [84]. Other functional network involving non coding and coding RNAs have been reported e.g. in breast cancer [85, 86], CRC [87], gastric cancer [88] and NSCLC [89].

Here we describe the most relevant methods developed to investigate the ncRNAs interactome, for example, dCHIRP (domain specific chromatin isolation by RNA purification) is a method for simultaneous mapping of RNA-RNA, RNA-DNA and RNA-protein interactions at single domain level [90]. We classified these methods on the basis of the interactors and on the technical approach.

### Detection of RNA-RNA interaction

The interaction between two RNAs (inter-molecular) or between different regions of the same RNA molecule (intra-molecular) are one of mechanisms of the regulatory action of ncRNAs. Since computational methods can provide just a prediction of RNA-RNA interaction (RRI), different low and high- throughput methods have been developed to directly solve these molecular events [91].

#### Low-throughput techniques

RRI may be directly investigated through low-throughput biophysical and biochemical methods, such as electrophoretic mobility shift assay (EMSA), surface plasmon resonance (SPR) or single molecule forster resonance energy transfer (FRET). In EMSA, RNA fragments are extracted from cells and RRI is evaluated through electrophoresis based on molecular mass (larger in the case of interaction) [92]. In SPR, RRI is detected in real time through the immobilization of one RNA fragment on a sensor by streptavidin-biotin [93]. In FRET, the fragment is immobilized on quartz surface and the real time monitoring is based on the interaction of two fluorescent dyes in a closed space. These methods are not able to identify the precise region of the interaction. An example of the application of RRI techniques has been provided by Tianyou Liu et al., which characterized lncRNA DLEU1 in the context of CRC progression, and found by EMSA that DLEU1 directly binds SMARCA1 [94].

#### High-throughput targeted techniques

NGS technologies have been applied to investigate RRI at transcriptomic level. Among them, we mention *i)* crosslinking, ligation and sequencing hybrid (CLASH) and *ii)* hybrid and individual-nucleotide resolution ultraviolet cross-linking and Immunoprecipitation (HiCLIP RNA), which are able to identify duplex of two ligated RNAs, *iii)* RNA interactome analysis followed by deep sequencing (RIA-seq) and *iv)* RNA antisense purification and sequencing (RAP-seq) that explore the interactome for a target RNA. For example, Helwak et al. mapped the human miRNA interactome by CLASH and revealed non-canonical binding sites [95].

#### Transcriptome-wide techniques

The last frontier for RRI detection techniques is based on sequencing-based methods at transcriptome-wide level. *i)* psoralen analysis of RNA interactions and structures (PARIS) [96], *ii)* sequencing of psoralen crosslinked, ligated, and selected hybrids (SPLASH) [97] and *iii)* ligation of interacting RNA followed by high-throughput sequencing (LIGR-seq) [98] are three methods which differs in the isolation and enrichment of RNA-RNA duplex but all rely on cross-linking of RNAs, ligation of duplexes and high-throughput sequencing. These techniques allow the identification of all types of RRI, included unknown interactors and unexplored regions that can be mapped at high resolution.

### Study of RNA- chromatin interaction: hybridization-based methods

To investigate lncRNAs binding sites on chromatin *i)* Chromatin isolation by RNA purification (ChIRP) *ii)* RNA antisense purification (RAP) and *iii)* capture hybridization analysis of RNA targets (CHART) are the most common experimental approaches [99]. *i)* ChIRP is a technology that enables the analysis of lncRNA-DNA complexes by the extraction of chromatin from cross-linked cultured cells, sonication, hybridization with biotinylated oligos and separation with magnetic streptavidin beads [100]. The output of the analysis depends from the method used, from the wet lab techniques, such as real-time PCR to the more recent and high-throughput methodologies, such as ChIRP-seq. *ii)* RAP differs from ChIRP for the use of longer antisense RNA probes with enhanced affinity to the target lncRNA. The products isolated with this method could undergo NGS analysis. *iii)* CHART similarly to ChIRP and RAP involves the purification of cross-linked RNA, DNA and proteins complexes, but differs for the use of short affinity-tagged oligonucleotides targeted to the region of predicted lncRNAs open binding sites [101]. An example of the application of hybridization-based approaches has been provided by Megan E. Forrest et al. who demonstrated by ChIRP-Seq the direct association of the colon cancer-upregulated lincDUSP with genes implicated in the replication-associated DNA damage response and in cell-cycle control [102].

### Analysis of RNA-protein interaction

lncRNAs may interact with RNA-binding proteins (RBPs) to play their regulatory roles. Immunoprecipitation and affinity-based approaches have been developed to identify proteins involved in the functional complexes.

#### Immunoprecipitation-based methods

RNA Immunoprecipitation (RIP) is the most frequently used method to study lncRNA-protein interaction and is based on the immunoprecipitation of the complex by the use of an antibody directed to a target protein. After purification, lncRNAs can be analyzed through PCR, microarray (RIP-Chip) or NGS (RIP-seq) [103]. Subsequently, the method has been improved to map the precise binding sites, for example cross-linking and Immunoprecipitation (CLIP) differs from RIP in the use of UV radiation to cross-link RNA and binding proteins allowing stringent purification condition. In the last years, CLIP has been combined with other techniques such as NGS (CLIP-Seq) [104] and further modified to improve cross-linking efficiency and sequence read resolution (Photoactivatable ribonucleotide-enhanced cross-linking and immunoprecipitation: PAR-CLIP) [105]. Krell J et al. combined RIP-seq and PAR-CLIP-Seq to identify the precise binding site between AGO2-bound miRNAs and their mRNA targets, by determining the control of AGO2 loading by TP53 as a novel miRNA-mediated mechanism in cancer development [106].

However, CLIP or RIP are applicable only if an antibody against a specific protein is available. To overcome this limit, different approaches have been developed, such as RNA-tagging [107], or Targets of RNA-binding proteins Identified By Editing (TRIBE-seq) [108], which are able to detect and analyze protein-RNA interaction in vivo independently of a specific antibody, by using fusion proteins which bind the target RNAs.

#### Affinity-based methods

To move towards the identification of RNA interactors at the proteomic level, the best approach is Biotinylated RNA-protein pull-down followed by liquid chromatography-mass spectrometry/mass spectrometry (LC–MS/MS). In this method, target RNA is synthesized, labeled with biotinylated uridines, incubated with cellular lysates, pulled-down with streptavidin beads and finally, the RNA-binding protein complexes are separated through Sodium Dodecyl Sulphate - PolyAcrylamide Gel Electrophoresis (SDS-PAGE) and analyzed through MS. Anbang Wang et al. demonstrated through this technique that the lncRNA EGFR-AS1 interact with HuR, which affects mRNA stability of EGFR by promoting cell growth and metastasis in renal cancer [109]. However, in the last years, many approaches have been described to increase specificity or sensitivity such as ChIRP-MS [110].

## Promising approaches for therapeutic intervention

The deregulation of ncRNAs in cancer cells, in term of expression profiling, interactome, as well as other intrinsic changes promoting tumor formation, offers the rational to consider them as a class of potential therapeutic targets. Given the diversity in their potential mode of action, several types of genomic and functional approaches have been developed to directly or indirectly target ncRNAs depending on whether they are oncogenes to be inhibited or tumor suppressors to be replaced. Among them we discuss about *i)* post-transcriptional RNA degradation using small interfering RNA (siRNAs) or synthetic antisense oligonucleotides (ASOs); *ii)* modulation of ncRNA genes by using genome-editing techniques; *iii)* replacement of ncRNAs; *iv)* inhibition of RNA–protein interactions or preventing secondary structure formation by using small molecules. We report several references of preclinical studies which highlight the power of these techniques in functional investigation. However, despite all these approaches are promising as therapeutics interventions, many barriers, for example in delivery systems, need to be overcome in the vision of their clinical translation.

### ncRNAs targeting: ASOs

ASOs are synthetic nucleic acids sequences that binds, via Watson-Crick base pairing, to complementary RNA substrates. The two mechanisms of action of ASOs are the recruitment of RNase H to the DNA–RNA heteroduplex to degrade RNA [111] or the inhibition of biogenesis or translation [112]. Through chemical alterations of the natural nucleotides, ASOs have been designed to retain drug-like properties. The phosphorothioate modification of the linkage leads to ASOs protection from degradation by nucleases and to increase half-life in serum, while still supporting RNase H activities. These so-called first-generation ASOs composed solely of deoxy residues were limited in clinics. Second generation ASOs contain a central region of about 10 phosphorothioate DNA nucleotides flanked by nucleotides modified at the sugar (“gapmer” design). Third generation ASOs are instead composed from LNA modified antisense oligonucleotides gapmers which are enriched with LNA in the flanking regions and DNA in a LNA-free central gap. LNAs are nucleic acid analogs in which the ribose ring is “locked” by a methylene bridge between the 2′ oxygen and the 4′ carbon. A representativstudy about the use of ASOs for functional ncRNAs validation has been reported from Amodio et al., who demonstrated that the inhibition of lncRNA MALAT1 by a LNA-gapmeR antisense oligonucleotide, antagonizes cell proliferation and triggers apoptosis both in multiple myeloma cell lines and in a murine xenograft model [7]. The anti-multiple myeloma activity of miRNA-221 has been instead demonstrated through its inhibition in vitro and in vivo mediated from a specific LNA-i-miR [113, 114].

### ncRNAs targeting: RNAi

RNA interference (RNAi) is an endogenous and well-conserved post-transcriptional modulation mechanism, which works through paring of endogenous or exogenous dsRNA with a target mRNA. Specifically, a dsRNA is firstly cleaved in a 21-RNA sequence, called siRNA, by Dicer and then is loaded in RISC (RNA induced silencing complex), which is located in cytosol. Here the passenger strand is discarded, the guide strand is paired with target mRNA and, depending on complementarity, silencing is induced through degradation or translational repression [115, 116]. This physiological mechanism has been frequently applied experimentally for therapeutic task in molecular oncology and then modified to perform high throughput screening by using pools of siRNAs. As matter of fact, several libraries targeting miRNAs and lncRNAs have been developed and led to the identification of ncRNAs affecting drug response or cancer pathways [116]. For example, the use of genome wide miRNA libraries allowed *i)* the discovery of miR 195 synergic role in microtubule targeting agent response in lung cancer [117] *ii)* the identification of several miRNAs relevant in trastuzumab resistance in HER2 positive cells [118] *iii)* the discovery of miRNAs determining navitoclax susceptibility in CRC cell lines [119]. The application of high-throughput siRNA-based screening targeting lncRNAs clarified the oncogenic role of linc0015226 and an unprecedented reported role of DRAIC in autophagy regulation in breast cancer cells [120]. On the other hands, synthetic siRNAs has been also used as therapeutic tools inducing ncRNA degradation. For example, a siRNA-mediated HOTAIR degradation suggested a therapeutic role of HOTAIR inhibition, since its negative regulation reduced tumor cells dissemination in an in vitro breast cancer model [67]. Moreover, a siRNA-based inhibition of MALAT1 suggested its critical role in temozolomide resistance in glioblastoma multiforme, since its inhibition restored drug sensitivity attenuating cancer stem cells stemness and proliferation [121].

### CRISPR-Cas9 ncRNAs genomic editing

In the past 10 years, several methods for genome editing have been developed such as Zinc-finger nucleases (ZFNs), transcription activator like effector nucleases (TALENs) and clustered regularly interspaced short palindromic repeats (CRISPR)-associated nuclease 9 (CRISPR/Cas9) [122]. Here, we focus on CRISPR/Cas9 system, which represents the last revolution in biological research, especially for ncRNAs study. This system works as a molecular “scissor” and has been developed by modifying the adaptive prokaryotic immune system in order to induce a well-defined genetic change in eukaryotic cells through a “guide RNA” and Cas9 protein. The guide RNA (gRNA) is 20 nucleotides in length and is homologous to a specific region of the target DNA flanking a 3 DNA base pair protospacer adjacent motif (PAM)-sequence recognized from the Cas9, which is an endonuclease able to induce a double stranded break (DSB). The Cas9-mediated DSB may be repaired by non-homologous end joining (NHEJ) by inducing non-in frame small insertion or deletions that disrupts the targeted locus (knock-out (KO) approach), or by homology directed repair (HDR) in the case of a donor DNA is supplied to insert a desired sequence (knock-in) [123]. Several validation studies have been performed through this strategy to investigate the function of selected lncRNAs or miRNAs in solid and hematological malignancies [124–126]. For example, through the CRISPR-Cas9 system, the roles of *i)* LncRoR as activator of MAPK/ERK pathway [127], *ii)* LncAK023948 as positive regulator in Akt pathway [128] and *iii)* LncBC200 as promoter of cell growth have been demonstrated in breast cancer [129]. CRISPR-Cas9 approach has been also used to reduce the expression of miRNAs up to 96% in vitro and in vivo by targeting the miRNAs biogenesis site. This KO approach resulted more robust, precise and stable respect than other techniques available for loss of function studies (such as antisense inhibitors) [130]. Different applications of CRISPR-Cas9 system also provided the possibility to disclose the oncosuppressive role of miR-210 in renal cell carcinoma cell lines [131] and of miRNA182-5p in chronic myeloid leukemia [132]. Furthermore, several studies focused on the possible delivery strategies for the use of CRISPR-Cas9 system as technology for miRNA therapeutics [133, 134].

Considering the high impact of this technology on molecular studies [135], CRISPR-Cas9 system have been further modified to induce genetic changes increasingly precise and sophisticated, up to base editing level. At this aim, Cas9 protein has been fused to specific domains in order to work as stimulator or suppressor of genetic transcription (CRISPR-activation or CRISPR-interference system, respectively) [136–139] and to induce transient loss of function (LOF) or gain of function (GOF).

Moreover, the last progress in this context is represented from the use of CRISPR-Cas9 pooled library, which consist in thousands of plasmids encoding for multiple barcoded gRNAs targeting different genes simultaneously, with a strong reduction of time and costs related to functional validation experiments [140]. A representative study of CRISPR-interference based screening has been performed by Liu et al. in 7 transformed cell lines by targeting ~ 16.000 lncRNAs. They identified 499 lncRNA loci involved in cellular growth and tissue specific transcriptional regulation [141]. Kurata et al. identified cell fitness-associated miRNAs with a miRNA-based CRISPR-Cas9 pooled library targeting ~ 1600 annotated human miRNA stem-loops [142]. By using a genome wide CRISPR-Cas9 LOF screen, Wallace et al. identified miRNAs involved in myeloid leukemia cell growth, of which miR-155 was the top candidate [143]. Moreover, CRISPR/Cas9-based synergistic activation mediator (SAM) system revealed the role of lncRNA AK023948 as positive regulator of AKT in breast cancer [128]. A genome-scale deletion screen of ~ 12.000 lncRNAs through a paired-guide RNA pooled library allowed the identification of 51 lncRNAs involved in a positive or negative regulation of tumor growth [144]. The major limit of this technology is represented by off-target effects, even though several approaches are going to be applied to overcome or at least reduce this important issue [145, 146]. For what concerns clinical translation, CRISPR-Cas9-based approaches are still in its infancy, especially because of the eventuality of adverse immune response due to bacterial Cas9, generally delivered by viral vectors, and because of ethical issues intrinsic to genome editing applications in human [123].

### ncRNAs replacement

Many relevant ncRNAs in cancer are genomically deleted or downregulated acting as tumor suppressors, whereby their reactivation may have anticancer activity. Replacement strategies are widely applied to restore the functionality of tumor suppressor miRNAs using double-stranded RNA of 22-mer oligonucleotides sharing the same sequence of mature miRNA or its precursor, and for this reason they are known as *mimics*. A well known example is the replacement of miR-34a, a tumor suppressor that is lost or expressed at reduced levels in a broad range of tumor types [147]. The exogenous introduction of miR-34a mimics in vitro showed inhibition of cell proliferation, migration and invasion, alone or in combo with anticancer therapies [148]. These results have lead to the first clinical application of a liposomal formulation of miR-34a mimic (MIRX34) in clinics [149]. Another approach is the use of synthetic RNA molecules able to mimic hairpin structures of lncRNAs. An example is GAS5, a lncRNA that acts as a decoy for the glucocorticoid receptor (GCR) blocking the transcription of target genes [150]. To overcome GAS5 loss of function due to acquired mutations in the GCR response element sequence, Pickard et al. reported the generation of an oligonucleotide that mimic the mutated region sequence on breast cancer cells showing pro-apoptotic activity similar to wild-type GAS5 [151].

### Limitation of RNA-based therapies

The reactivation of tumor suppressor ncRNAs as well as the use of nucleic acids-based methods requires the availability of efficient in vivo delivery systems to overcome biological drawbacks associated with such strategies. A first barrier is the transport across the cell membranes limited to diffusion of small and relatively hydrophobic compounds. In addition, RNA molecules show short half-life in vivo environments due to the highly risk of degradation by cellular nuclease such exonuclease or endonuclease. An important issue is also the activation of innate immune response to foreign RNAs through toll-like receptor and retinoic acid inducible gene I protein pathways. This results in the production of type 1 interferon and subsequent release of inflammation associated cytokines. Finally, it is important to avoid, or at least predict and recognize, off-target effects and to reduce the toxicity. At this aim siRNA and ASOs as well as ncRNAs can be encapsulated inside lipid-based nanoparticles in order to ensure its survival against biological agents and delivered into cancer cells, also in a target specific manner. In addition, the development of N-acetylgalactosamide (GalNAc) conjugated to siRNAs has enhanced hepatic uptake [152]. To extend delivery to other tissues, alternative conjugation methods including lipids such as cholesterol, peptide nucleic acids (PNAs), and antibodies have been used.

### Small molecules

Although the RNA therapeutics research is mainly focused on oligonucleotides, the application of SMs to target specific ncRNAs have emerged as a feasible and efficient strategy and may in part overcome limitation of RNA approaches based on Watson and Crick hybridization. Computational biology can allow the identification, prediction of docking sites and design of these SMs, as we mentioned above. Moreover, the advantages of SMs are their chemical nature that make them suitable for conventional drug development. In contrast, limitations are poor specificity and complex design compared with sequence-specific methods. SMs exert their therapeutic effect on ncRNAs by specific binding to secondary or tertiary structures as miRNA hairpin precursors or structural elements of lncRNAs such as the triple-helical structure of MALAT1 and NEAT1. In this way, SMs can destabilize the transcript or allosterically interfere with the interaction between the RNA and its protein partners. An additional mechanism of action of SMs is the binding to the Dicer or Drosha nuclease processing sites, which could affect the biogenesis of miRNAs. The development of bioinformatics tools allowed to perform high-throughput screening of ncRNA libraries against datasets of small molecules identifying strong interactions. Using this strategy Li et al. tested the ability of targaprimir-96, a bleomycin A5 conjugate, to target pri-miR-96. This compound directly block pri-miR-96 maturation via Drosha leading to the upregulation of miR-96 target FOXO1 and the induction of apoptosis in breast cancer cells [153]. Similarly, Haga et al. showed that inhibition of Dicer cleavage sites in pre-miR-544 resulting in sensitization of breast cancer cells to hypoxic stress [154].

## From bench to bedside: ncRNAs in clinical practice, promise or challenge?

As we discussed above, numerous preclinical studies are focusing on ncRNAs characterization with the aim to clarify their role in tumorigenesis and to disclose their contribution for diagnostic, prognostic and therapeutic purposes. We reported several strategies, which emphasized the promising use of ncRNAs for cancer treatment. Now, we discuss about the bench to bedside translation of the ncRNAs therapeutics in the ongoing clinical trials. MiRNAs are the most extensively studied as both therapeutic candidates or targets [155, 156], followed by lncRNAs, which are emerging in the clinical setting [157–161].

For example, it is noteworthy that ncRNAs may play a crucial role in chemo and radio resistance, which is the major challenge of current anticancer treatments [162, 163].

On https://clinicaltrials.gov website are reported 304 studies involving miRNAs in clinical applications, of which 101 are interventional studies at different phases. Among them, we mention the phase I clinical trial NCT02369198 based on the administration of TargomiRs as 2nd or 3rd line treatment for patients with recurrent malignant pleural mesothelioma and NSCLC. This drug consists in a miR-16-based microRNA mimic, nanoparticles for delivery and an anti-EGFR bispecific antibody. Moreover 13 studies are reported concerning lncRNAs, of which 11 are observational and 3 interventional (NCT02641847 phase I/II, NCT02221999 phase II/III and NCT03000764 -phase not applicable-). However, in the majority of cases, miRNAs and lncRNAs are evaluated only in term of expression profiling to validate them as biomarkers, while RNA-based therapeutics or SMs are not yet clinical interventions under widespread investigation. This points the need to work hard to translate the large and promising preclinical studies in early clinical trials, This scenario strongly indicates the need of highly multidisciplinary efforts to make “dark matter” a major mean in the fight against cancer in the next future.

## Conclusion

Here we have reviewed research strategies aimed to investigate the role of miRNAs and lncRNAs in cancer. The availability of new powerful sequencing and molecular technologies allowed the overcoming of several potential caveats, such as the low abundance of ncRNAs, the subcellular spatial localization and their instability. Improvements in wet laboratory techniques together with in silico tools significantly improved the knowledge of the “dark matter” of the genome in terms of discovery, annotation and functional validation. Apart from the most widely adopted methods that we have described, other strategies have emerged to improve the global characterization of ncRNAs in the last 10 years (Table 2) and the optimization of these methods is still ongoing. Notwithstanding, in some cases, it is not possible to completely clarify the function of non-coding transcripts out of a physiological context, especially because are poorly conserved between species, making the in vivo experiments not easily translatable for applications in humans and because, if compared to coding genes, are more difficult to be explored. A lot of novel ncRNAs are completely uncharacterized by making more complex the understanding of their role. In addition, for the majority of lncRNAs, crystallographic structures leading the design of SMs are still unknown. Moreover, despite the rapid evolution of ncRNAs targeting methods (ASOs, SMs, etc) provides an exciting rationale for clinical applications, several obstacles still stand in the way, such as delivery strategies, stability, specificity and toxicity of the treatments. Further advances in the next future are expected to better clarify the regulatory network behind ncRNAs perturbations, and mostly to move experimental results from bench to bedside.

**Table 2:** Summary table of methods that have been developed to globally investigate ncRNAs conformation, relative activity of sites undergoing transcription, or half-life

TECHNIQUE	BRIEF DESCRIPTION	REF.
SHAPE (Selective 20-hydroxyl analysed by primer extension)	Is a technique to unravel the secondary structure of lncRNAs	[164–166]
PARS (Parallel analysis of RNA structure)	Is a methods able to explore changes in lncRNAs structurome that can occurs in carcinogenesis, recently implemented with the Illumina platform (nextPARS) to provide results with higher throughput and sample multiplexing	[167–169]
Frag-Seq (Fragmentation sequencing)	Is an assay for probing RNA structure at transcriptome-wide level by combining RNA-seq and tools determining nuclease accessibility at single base resolution	[99, 170, 171]
ICE-seq (Inosine chemical erasing sequencing)	Is an approach able to reveal the deregulation that may occur in A-to-I editing of lncRNAs in cancer allowing relevant effect on their secondary structure and then, on the interaction with other RNA molecules	[168, 172, 173]
BRIC-seq (50-bromo-uridine immunoprecipitation chase–deep sequencing)	Is a method that determine precise RNA half life into cells in physiological and pathological conditions	[174–176]
FISSEQ (Fluorescent in situ sequencing)	Is a method, based on SOLiD sequencing, revealing spatial changes in lncRNAs during cancer	[99, 177, 178]
Gro-seq (Global run-on assay sequencing)	Is an NGS-based method that provide information about location, orientation and density of RNAs undergoing active transcription by RNA pol II.	[174, 179, 180]

## Data Availability

Not applicable**.**

## Abbreviations

ncRNAs: Non-Coding RNAs
miRNAs: MicroRNAs
lncRNAs: Long Non Coding RNAs
NGS: Next Generation Sequencing
IVT: *InVitro* Transcription
SAGE: Serial Analysis of Gene Expression
RNA-seq: RNA Sequencing
CRC: Colorectal Cancer
DP-seq: Designed Primer-based Sequencing
CAGE: Cap Analysis Gene Expression
TSS: Transcription Start Sites
NSCLC: Non-Small Cell Lung Cancer
MFE: Minimal Folding Energy
HMM: Hidden Markov Model
SCFG: Stochastic Context Free Grammar
SMs: Small Molecules
NB: Northern Blot
RT-qPCR: Reverse Transcription Quantitative PCR
ISH: In Situ Hybridization
FISH: Fluorescence In Situ Hybridization
DIG: Digoxigenin
LNA: Locked Nucleic Acid
RRI: RNA-RNA Interaction
EMSA: Electrophoretic Mobility Shift Assay
SPR: Surface Plasmon Resonance
FRET: Forster Resonance Energy Transfer
CLASH: Crosslinking, Ligation and Sequencing Hybrid
HiCLIP: Hybrid and Individual-Nucleotide Resolution Ultraviolet Cross-Linking and Immunoprecipitation
RIA-seq: RNA Interactome Analysis Followed by Sequencing
RAP-seq: RNA Antisense Purification and Sequencing
PARIS: Psoralen Analysis of RNA Interactions and Structures
SPLASH: Sequencing of Psoralen Crosslinked, Ligated, and Selected Hybrids
LIGR-seq: Ligation of Interacting RNA followed by Sequencing
ChIRP: Chromatin Isolation by RNA Purification
RAP: RNA Antisense Purification
CHART: Capture Hybridization Analysis of RNA targets
RBPs: RNA-Binding Proteins
RIP: RNA Immunoprecipitation
CLIP: Cross-Linking and Immunoprecipitation
PAR-CLIP: Photoactivatable Ribonucleotide-Enhanced Cross-Linking and Immunoprecipitation
TRIBE-seq: Targets of RNA-Binding Proteins Identified By Editing followed by Sequencing
LC–MS/MS: Liquid chromatography-Mass Spectrometry/Mass Spectrometry
SDS-PAGE: Sodium Dodecyl Sulphate - PolyAcrylamide Gel Electrophoresis
SiRNAs: Small Interfering RNA
ASOs: Synthetic Antisense Oligonucleotides
RNAi: RNA Interference
RISC: RNA Induced Silencing Complex
ZFNs: Zinc-Finger Nucleases
TALENs: Transcription Activator Like Effector Nucleases
CRISPR: Clustered Regularly Interspaced Short Palindromic Repeats
gRNA: Guide RNA
PAM: Protospacer Adjacent Motif
DSB: Double Stranded Break
NHEJ: Non-Homologous End Joining
KO: Knock-Out
HDR: Homology Directed Repair
LOF: Loss Of Function
GOF: Gain Of Function
SAM: Synergistic Activation Mediator
GCR: Glucocorticoid Receptor
GalNAc: N-Acetylgalactosamide
PNAs: Peptide Nucleic Acids
PA: Public Available
